# Tumor Microenvironment in Oral Cancer Following Neoadjuvant Pembrolizumab: Preliminary Analysis of the Histopathologic Findings

This article has been retracted.

**DOI:** 10.3389/froh.2021.653104

**Published:** 2021-04-23

**Authors:** Alex Dobriyan, Iris Gluck, Eran Alon, Iris Barshack, Ran Yahalom, Marilena Vered

**Affiliations:** ^1^Department of Oral and Maxillofacial Surgery, The Chaim Sheba Medical Center, Tel Hashomer, Israel; ^2^Head and Neck Cancer Unit, The Chaim Sheba Medical Center, Institute of Oncology, Tel Hashomer, Israel; ^3^Sackler Faculty of Medicine, Tel Aviv University, Tel Aviv, Israel; ^4^Department of Otolaryngology—Head and Neck Surgery, The Chaim Sheba Medical Center, Tel Hashomer, Israel; ^5^The Chaim Sheba Medical Center, Institute of Pathology, Tel Hashomer, Israel; ^6^Department of Oral Pathology, Oral Medicine and Maxillofacial Imaging, School of Dentistry, Tel Aviv University, Tel Aviv, Israel

**Keywords:** oral squamous cell carcinoma, pembrolizumab, tumor microenviroment, immune reaction, cancer-associate fibroblasts

## Abstract

**Background:** The tumor microenvironment (TME) of oral squamous cell carcinoma (OSCC) is associated with immune suppression, one of the pathways being the programmed death receptor 1 (PD-1) and its ligands (PD-L1/PD-L2). Checkpoint inhibitors of PD-1/PD-L1, like pembrolizumab, have been recently approved for treatment of OSCC. We described the histologic findings in OSCC following neoadjuvant pembrolizumab, including identification of immune-related cell populations and cancer-associated fibroblasts (CAFs).

**Materials and Methods:** Patients with OSCC clinical stages 3 and 4 and a combined PD-L1 score >1 were randomized either to the standard oncologic protocol or to the pembrolizumab arm of MK-3475-689 study for Head and Neck, Lip, and Oral Cavity. The latter were given two standard doses of 200 mg of pembrolizumab, 3 weeks apart, and then underwent surgical oncologic procedure according to the initial stage. Sections from the resection specimens were analyzed for pathological response to pembrolizumab. Various populations of immune-related cells within the tumor microenvironment were characterized by immunohistochemistry, as were the CAFs.

**Results:** Three patients who were randomized to the pembrolizumab study were described. One patient presented with a tongue SCC, the other two had SCC of the mandibular ridge with bony involvement. Only the patient with tongue SCC showed clinical complete response. Microscopically, the tumor was replaced by a granulomatous type of inflammation. Immunohistochemical stains revealed massive T cell rich (CD3^+^) infiltrate, with approximately equal amounts of CD4^+^ and CD8^+^ cells, numerous macrophages of CD68^+^ and CD163^+^ phenotypes; no CAFs were identified. The other two patients were regarded as non-responders as at least 50% of the tumor was viable. The tumor microenvironment of these tumors was generally associated with a lesser extent of inflammatory response compared to the tongue tumor, a variable CD4^+^/CD8^+^ ratio and presence of CAFs. Neither T regulatory cells (FOXP3^+^) nor natural killer cells (CD56^+^, CD57^+^) were identified in any of the cases.

**Conclusion:** We showed that characterizing the specific populations of immune-related cells and CAFs after treatment with pembrolizumab, may add to our understanding of the tumor-TME interactions in this setting. These findings should be investigated in future studies on a larger number of patients.

## Introduction

Squamous cell carcinoma (SCC) is the most common histological type of cancer in the head and neck, with that of the oral cavity (OSCC) being the most commonly affected location in this area [1]. Annually, there are around 700,000 new cases of SCC in the head and neck region and 380,000 deaths due to disease worldwide [2]. The standard of care for resectable tumors includes surgical resection of the primary tumor and the regional draining lymph nodes, and adjuvant radiotherapy or chemotherapy, depending mainly on patient stage and resection margin status [3]. For the last four decades, across all stages of the disease and most countries, the 5-year survival rate has remained ~50% (excluding human papilloma virus- and Epstein-Barr virus-related SCCs) [2, 4]. The grim prognosis of the patients together with the serious and sometimes life-long side effects caused by current treatment modalities, the need to find novel treatment modalities for OSCC and other SCCs of the head and neck, has become imperative.

The tumor microenvironment (TME) is the complex milieu of non-malignant cells and extra-cellular matrix components that surrounds solid tumors and it is the reciprocity of TME-tumor relations that ultimately defines the malignant behavior [5]. The TME is regarded as a major mediator of immune suppression in many solid cancers [6–8]. One of the molecular pathways that leads to tumor immune escape is the abrogation of T lymphocyte cell activation, proliferation and anti-tumor response, via expression of programmed death receptor 1 (PD-1) on T cells and of PD-1 ligands (PD-L1/PD-L2) on the tumor cells [9, 10]. Therefore, the PD-1/PD-L1 pathway became a critical immune checkpoint used by TME-tumor “collaboration” to suppress anti-tumor immunity, but at the same time, it turned into a feasible target for the development of pharmacological agents aimed to inhibit zthe PD-1/PD-L1 interaction and restore the anti-tumoral response of the T cells. Pembrolizumab (MK-3475) is a potent, highly selective, humanized monoclonal antibody that prevents PD-1 binding with PD-L1 and PD-L2 [10].

The Society for Immunotherapy of Cancer recently published a consensus statement on pembrolizumab for the treatment of SCC of the head and neck, emphasizing that targeting proteins such as PD-1 and PD-L1 have shown promise of durable, long-term survival in responding patients [2]. Furthermore, in 2019, the Food and Drug Administration (FDA) approved pembrolizumab as a single agent for patients with head and neck SCC, whose tumors express a PD-L1 combined positive score ≥1, thus officializing the first immunotherapeutic modality regarding this group of cancers [2]. Nowadays, there are attempts to determine the molecular profile or genetic signature based on tumor tissue prior to administration of pembrolizumab, that could predict clinical responsiveness [10–14].

The use of pebrolizumab in oral cancer is relatively new and treatment outcomes have been primarily evaluated by clinical parameters of patients' survival. Histologic changes related to this modality have not been well-documented and usually addressed other types of SCC but not OSCC [15–17]. The present brief research aimed to report the histologic findings within the TME in a small series of patients with OSCC following neoadjuvant pembrolizumab. Furthermore, the variety of immune-related cell populations and presence of cancer-associated fibroblasts (CAFs) were immunohistochemically identified and discussed in the context of the importance of the tumor-TME interactions.

## Materials and Methods

During 2019–2020, 46 patients diagnosed with OSCC, clinical stages 3 and 4, in the Department of Oral and Maxillofacial Surgery, Chaim Sheba Medical Center, and a PD-L1 combined positive score >1 (https://www.agilent.com/cs/library/usermanuals/public/29314_22c3_pharmDx_hnscc_interpretation_manual_us.pdf) were presented with the possibility of entering the MK-3475-689 study for Head and Neck, Lip and Oral Cavity. Written informed consent was obtained from 16 patients, out of whom 11 were screened out, two were randomized for only surgery and three were randomized for neoadjuvant pembrolizumab (Keytruda; Merck, Kenilworth, NJ, USA) followed by surgery. The study is still enrolling patients; it has been approved by the IRB of the medical center #4622/4623-17-SMC.

According to the protocol, the patients in the pembrolizumab category received a standard dose of 200 mg, the first being administrated immediately during the day of randomization and the second dose 3 weeks after. This was followed by surgery that had to be performed in a total time-frame of 6 weeks ± 10 days from the day of randomization. The surgical oncologic protocol was tailored according to the initial stage status, irrespective of the extent of tumor responsiveness to the neoadjuvant agent. Post-operative need for adjuvant radiation/chemotherapy was decided according to pre-operative established patient stage and resection margin status. The continuation or discontinuation of pembrolizumab was defined by assessment of the tumor microscopic response. Unrelatedly to post-operative administration of pembrolizumab, follow-up protocol was planned as standard for patients with OSCC.

The resected specimens were formalin fixed and paraffin embedded. Each specimen was sampled so that sections represented distances between the tumor and each of the surgical inked margins. These sections were routinely stained by hematoxylin and eosin (HE) for diagnostic purposes. In addition, immunohistochemical stains were performed to define populations of immune-related cells. We also performed stains to identify cancer-associated fibroblasts (CAFs), a prominent component of the TME, that were found to upregulate expression of PD-L1 on tumor cells [1, 6, 18, 19]. In regard to immunohistochemical stains, the used antibodies by types, manufactures and staining procedures are detailed in Table 1. Results are described qualitatively.

**Table 1:** Antibodies used for identification of immune cells and cancer-associated fibroblasts.

**Primary Antibody**	**Targeted cell type**	**Manufacturer**	**Catalog #/Concentration**	**Positive control tissue**
AE1/AE3	Epithelium (normal, neoplastic)	Novocastra, Newcastle upon Tyne, UK	NCL-L-AE1-AE3/1:100	Tonsil
CD3	T lymphocytes	Dako, Glostrup, Denmark	A0452/1:100	Tonsil
CD4	T helper cells	Master Diagnostica, Granada Spain	MAD6000/D7 (ready to use)	Tonsil
CD8	T cytotoxic cells	Diagnostic BioSystems, Pleasanton, CA, USA	DBS-12MAB/1:50	Tonsil
CD20	B lymphocytes	Dako, Glostrup, Denmark	M0755/1:400	Tonsil
CD68	Macrophages	Dako, Glostrup, Denmark	M0876/1:50	Tonsil
CD163	Macrophages (anti-inflammatory)	Cell Marque, Rocklin, CA, USA	163M-16/1:80	Tonsil
CD56	NK lymphocytes	Novocastra, Newcastle upon Tyne, UK	NCL-L-CD56/1:50	Skeletal muscles
CD57	NK lymphocytes	Novocastra, Newcastle upon Tyne, UK	NCL-NK1 (ready to use)	Prostate
Foxp3	Regulatory T cells	Abcam, Cambridge, UK	Abcam 20034/1:50	Appendix
αSMA	Cancer-associated fibroblasts	Dako, Glostrup, Denmark	M-085101/1:1000	Appendix
Calponin	Cancer-associated fibroblasts	Dako, Glostrup, Denmark	M3556/1:200	Appendix

*All stains were performed using Ventana BenchMark Ultra immunostainers and protocols (Roche Tissue Diagnostics, Oro Valley, Arizona, USA). Brown diaminobenzidine (DAB) staining was used to visualize positively stained cells. Calibration of antibodies was performed according to manufacturers' instructions. Validation of calibration was performed on 10 known positive tissues and 10 known negative tissues, according to the guidelines of College of American Pathologists (CAP, available at: https://www.cap.org/protocols-and-guidelines)*.

## Results

In this study, we present the three patients who were randomized for the pembrolizumab arm of the study and completed the neoadjuvant protocol and surgical procedures. The clinical and histopathological findings are summarized below.

### Patient #1

A 61-year-old male patient presented with a tumor on the right lateral aspect of the tongue in April 2020. Incisional biopsy was performed and the diagnosis was a conventional well-differentiated OSCC (Figure 1A). Medical history was remarkable for hyperlipidemia and repair of the mitral and tricuspid valves 4 years previously; he was a non-smoker, non-drinker. Following clinical and imaging work-up, the patient was staged clinically as T3N0M0. Following two doses of pembrolizumab, no clinical tumor was visible or palpated; some superficial irregular in foldings were the only findings in the area where the tumor used to be. In June, he underwent right hemiglossectomy and ipsilateral neck dissection of levels I–IV, as was planned according to the initial stage. Tongue was reconstructed with a radial forearm free flap. Macroscopically, the resected specimen of the tongue measured 7 cm × 3.5 cm × 3.0 cm and findings conformed to the clinical observations. Examination of the HE-stained slides of the tongue tumor revealed complete response, with only a small epithelial projection with dysplasia being suspected for a focus of residual viable tumor. The entire tumor underwent disintegration with a granulomatous type of inflammation that was generated around the non-vital tumor residues. Resection margins were considered clean. The examination of the lymph nodes revealed no metastatic tumor.

**Figure 1:** Patient #1: Photomicrograph of the incisional biopsy, hematoxylin and eosin stain **(A)**; Photomicrographs from the resection specimen, hematoxylin and eosin stain **(B)**, and immunohistochemically stained sections: pan-cytokeratin (AE1/AE3) **(C)**, CD3 **(D)**, CD4 **(E)**, CD8 **(F)**, CD20 **(G)**, CD68 **(H)**, CD163 **(I)**, alpha smooth muscle actin (αSMA) **(J)**, calponin **(K)** (**A**: scale bar 500 μm, **B,C**: scale bar 1 mm, and **D–K:** scale bar 500 μm).

The original extent of infiltration of the tumor could be essentially mapped according to the distribution of the reactive granulomas (Figure 1B). The panel of immunohistochemical stains is illustrated in Figures 1C–K. Pan-cytokeratin immunostain highlighted residual non-vital tumor cells within the granulomas. T lymphocytes (CD3^+^) were the most common type of immune cells. They were seen not only in association with the granulomatous reaction, but also accumulated at the interface and infiltrated into the oral lining epithelium, which morphologically showed only hyperplasia and hyperkeratosis, with no overt signs of dysplasia. This epithelium was in the area of the original tumor. A further sub-classification of the T lymphocytes showed that there were both CD4^+^ and CD8^+^ cells in about equal amounts and a similar distribution. B lymphocytes (CD20^+^) were remarkably less frequent than T lymphocytes and were mainly seen in association with the granulomatous inflammation, with only focal interface presence. Macrophages (CD68^+^) constituted a major part of the inflammatory cells of the granulomas, both the mono- and multi-nuclear giant cells. Their presence at the interface zone was only mild. On the contrary, macrophages identified as M2 type (CD163^+^), considered as acting in an anti-inflammatory/pro-tumoral mode [6], were mainly seen at the interface and encroached on the oral epithelium. They were also dispersed throughout the microenvironment and also constituted part of the immune cells within the granulomas, however the multinuclear giant cells were identified as CD163^−^. FOXP3, CD56- and CD57-stained cells were not identified. CAFs with alpha smooth muscle actin (αSMA)^+^ phenotype were absent, however spindle-shaped, CAF-like cells with a calponin^+^ phenotype, were occasionally seen in short intersecting bundles within the microenvironment.

The patient completed a full adjuvant radiotherapy course (66 Gy) by the end of October 2020. By mid-November 2020, he underwent the first post-operative PET-CT and was free of disease. He will complete pembrolizumab treatment for 15 cycles, every 3 weeks, according to the study protocol.

### Patient #2

A 61-year-old male was diagnosed with OSCC of the left mandible in August 2020. The incisional biopsy revealed a tumor of varying differentiation grades, ranging from well-differentiated areas with keratin formation and mild cellular atypia, to areas with keratin formation and remarkable cellular atypia, and to areas of poor differentiation (Figure 2A). Medical history was remarkable only for hypertension. The patient was a non-drinker, but used to smoke about one cigarette per day and one cigar twice a month for at least 10 years. Clinical stage was established as T4aN3bM0. On October, following 2 doses of pembrolizumab, the patient underwent segmental mandibulectomy and ipsilateral modified radical neck dissection (levels I–V). Mandible was reconstructed with immediate fibula free flap. Macroscopically, the specimen was a composite resection of the oral soft tissues, mandibular bone and overlying skin, measuring 10 cm × 9 cm × 6 cm.

**Figure 2:** Patient #2: Photomicrograph of the incisional biopsy, hematoxylin, and eosin stain **(A)**; Photomicrographs from the resection specimen, hematoxylin, and eosin stain **(B)**, and immunohistochemically stained sections: pan-cytokeratin (AE1/AE3) **(C)**, CD3 **(D)**, CD4 **(E)**, CD8 **(F)**, CD20 **(G)**, CD68 **(H)**, CD163 **(I)**, alpha smooth muscle actin (αSMA) **(J)**, calponin **(K)** (**A**: scale bar 100 μm, **B–K**: scale bar 200 μm).

Microscopically, examination of the HE-stained slides of the resected specimen revealed only partial response, with at least 50% viable tumor. There were morphological and cytological changes, probably therapy-related. These included cystic degeneration with minimal necrotic areas, cellular dis-cohesion, and apoptotic-looking tumor cells admixed with hemorrhagic and/or fibrotic areas (Figure 2B). Lymphocytic inflammatory infiltrate at the interphase with the residual vital tumor/partially disintegrated tumor was less compared to patient #1, but still tumor-infiltrating lymphocytes were readily present. Macrophages and foam cells were notable. Resection margins of both the soft and bony tissues were clean (>5 mm distance to the surgical margins). Examination of the neck dissection, revealed two metastatic lymph nodes, one with extra-capsular extension.

The panel of immunohistochemical stains is illustrated in Figures 2C–K. The residual tumor was highlighted by pan-cytokeratin immunostain. Among the inflammatory cells, T lymphocytes (CD3^+^) showed a considerable amount and usually surrounded the tumor. Among them, CD4^+^ cells were remarkably more frequent than CD8^+^ cells. B lymphocytes (CD20^+^) constituted only a minority of the immune response. Macrophages (CD68^+^) were abundant at the tumor-microenvironment interface; CD163^+^ macrophages were also present in a similar pattern as the CD68^+^ macrophages, but seemed to be less. FOXP3, CD56-, and CD57-stained cells were not identified. CAFs of αSMA^+^ phenotype were absent and CAF-like-calponin^+^ cells were present in a focal pattern.

By the end of December 2020, the patient completed a full adjuvant radiotherapy course (66 Gy) fortified with two courses of cis-platinum (100 mg/m^2^, every 21 days during radiation). As the response to pembrolizumab was not satisfactory, post-operative drug administration was discontinued. The patient has entered the routine follow-up protocol.

### Patient #3

A 67-year-old male was diagnosed with OSCC of the right mandible in June 2019. The incisional biopsy revealed a tumor that was moderately-to-poorly differentiated, with occasional central areas of commedo-like necrosis (Figure 3A). Medical history was remarkable for a non-small cell lung carcinoma of the right lung (2003) and left lung (2004). The patient was a non-drinker but a heavy smoker with a smoking history of 75-pack-years; he quit smoking upon diagnosis of the lung tumors. Clinical stage of the oral tumor was assessed as T4aN2bM0. Following two courses of pembrolizmab, he underwent segmental mandibulectomy and ipsilateral modified radical neck dissection (levels I-V). Mandible was reconstructed with immediate fibula free flap. Macroscopically, the resected specimen measured 8 cm × 6 cm × 3 cm.

**Figure 3:** Patient #3: Photomicrograph of the incisional biopsy, hematoxylin, and eosin stain **(A)**; Photomicrographs from the resection specimen, hematoxylin, and eosin stain **(B)**, and immunohistochemically stained sections: pan-cytokeratin (AE1/AE3) **(C)**, CD3 **(D)**, CD4 **(E)**, CD8 **(F)**, CD20 **(G)**, CD68 **(H)**, alpha smooth muscle actin (αSMA) **(I)**, calponin **(J)** (**A**: scale bar 100 μm and **B–J**: scale bar 200 μm).

Microscopically, examination of the HE-stained slides of the resection specimen revealed only about 50% response. Alongside with the vital residual tumor, there were tumor islands with central commedo-like necrosis, foci of entirely necrotic tumor and a moderate number of foreign-body granulomas in association with residual tumor cells (Figure 3B). Overall, there was a mild-to-moderate number of inflammatory cells (especially referring to lymphocytes) at the tumor-TME interface and within the tumor microenvironment. Resection margins of both the soft and bony tissues were clean (> 5 mm distance to the surgical margins). Examination of the neck dissection, revealed two metastatic nodes, one with entirely vital tumor and one with partially necrotic tumor. None of the involved nodes showed extracapsular extension.

The panel of immunohistochemical stains is illustrated in Figures 3C–J. The residual tumor was highlighted by pan-cytokeratin immunostain. T lymphocytes (CD3+) were seen surrounding the tumor islands however their presence was less impressive compared to patients # 1 and 2, and they tended to show a rather patchy or discontinuous distribution. Among them, CD8^+^ cells were remarkably more frequent than CD4^+^ cells. B lymphocytes (CD20^+^) were considerably less frequent than T lymphocytes. Macrophages (CD68^+^) were readily seen mainly at the periphery of the necrotic tumor. FOXP3, CD56-, and CD57-stained cells were not identified. CAFs of αSMA^+^ phenotype were quite obvious surrounding part of the tumor foci, however, those CAF-like-calponin^+^ cells were scarce-to-absent.

The patient completed a full adjuvant radiotherapy course (66 Gy). As the response to pembrolizumab was not satisfactory, post-operative drug administration was discontinued. At the last follow-up examination by the end of November 2020, 1 year and 3 months post-operative, he was free of disease.

## Discussion

There is a growing body of literature demonstrating the clinical efficacy of pembrolizumab in the treatment of different types of solid cancers, including head and neck/OSCC. On a biological level, it is expected to find infiltration of the tumor by a remarkable lymphocytic reaction. This has been documented in only a few studies regarding SCC of the skin and non-small cell lung carcinoma (SCC type) and melanoma [15–17, 20]. Here, we describe a small series of patients with advanced OSCC (one tongue and two mandibular bone), who based on the combined PD-L1 score of >1, were eligible for neoadjuvant treatment with pembrolizumab and were assumedly expected to respond favorably. The clinical outcomes showed a complete response only for the tongue SCC. We provide a first detailed description of the histological findings observed in the resected tumors following two standard doses of pembrolizumab, with emphasis on the immunohistochemical characterization of the sub-types of immune-related cells within the TME.

Standardized assessment of the histologic changes following immune checkpoint blockade with neoadjuvant pembrolizumab has not been established so far. However, an initial assessment system has been attempted, aiming to provide a setting for studying the tissue-based outcomes of the drug mechanism of action [15]. This included parameters such as presence/absence of immune exclusion areas in the peri-tumoral stroma (i.e., areas devoid of lymphocytic infiltrates), dense immune infiltrates with features of activation (i.e., tertiary lymphoid structure, TLS), mature or proliferative (new) fibrosis, cholesterol clefts, and others. In our small series, we found a variable extend of inflammatory infiltrate within the TME, and it seemed that the case with the most abundant infiltrate was related to a complete pathological response (patient #1, tongue tumor), while a less conspicuous inflammatory process was related to a non-satisfactory response (patients #2 and 3, mandibular tumors). The extensive granulomatous type of inflammation was seen in the responsive patient (#1) and to a lesser extent in the other two patients. This type of inflammation was also reported in a responsive case of cutaneous SCC [16]. The incidence of these histological parameters should be further examined in larger groups of OSCC patients treated with pembrolizumab in order to find out any potential associations with clinical outcomes. Other factors are being investigated as potential indicators for the clinical benefit of pembrolizumab. One such factor is the baseline tumor size, which was found to be associated with treatment responsiveness in non-small cell lung cancer and melanoma [21]. Therefore, it seems that similar studies should also be performed in OSCC patients treated with pembrolizumab when more clinical data will be collected. Furthermore, examining the data as a factor of the location of the oral tumors in the soft tissues of the oral cavity vs. jawbones may potentially add important treatment planning considerations.

Focusing only on the general assessment of inflammatory response and on the presence of the cytotoxic T lymphocytes (CD8^+^) in pembrolizumab post-treatment specimens might not provide the entire landscape of immune-related modifications and other changes in the TME. We have already shown that the mere assessment of the extent of inflammation in the TME of OSCC was not by itself powerful enough to indicate clinical outcomes, but more specifically the extent of pro-tumorigenic immune cells [e.g., regulatory T cells (Tregs, FOXP3^+^) and tumor-associated macrophages (TAM2, CD163^+^)] were key features in determining patients' prognosis [22]. In the TME of pembrolizumab-treated tumors we presently showed not only varying amounts of CD3^+^ T cells, but a different CD4^+^/CD8^+^ ratio and variable amounts of macrophages with a different CD68^+^/CD163^+^ ratio. The impact of these variations on the efficacy of immune-related checkpoint inhibitors remains to be evaluated in larger samples.

CAFs, the major component of TME, have been shown to play a key-role in creating the immune-suppression milieu [5–8]. CAFs have the ability to inhibit T cell proliferation and differentiation and to upregulate expression of PD-L1 on the tumor cells, thus leading to T cell exhaustion, driving polarization of macrophages toward a pro-tumorigenic phenotype (CD163^+^), and encouraging the influx of T regulatory cells (FOXP3^+^) and other myeloid-derived suppressor cells. In addition, CAFs form a physical barrier between the tumor and the inflammatory infiltrate, termed as immune excluded zone, whereby the cytotoxic T cells are restricted to the periphery of the tumor, thus being sequestered from accessing the tumor. In the histological sections from patient #1 we showed a massive reaction of T lymphocytes with maximal direct physical interaction toward the oral epithelium in the area where the original tumor had been located, in parallel to absence of CAFs. In contrast, in patient #3, αSMA^+^ CAFs were located at the interface of tumor-TME in parallel to a moderate and patchy T cell reaction, which seem to support the paradigm of “CAFs in, T cells out.” However, not all CAFs are equal, and some subsets are believed to activate anti-tumor immune response [6, 8]. The finding of different combinations of CAF/CAF-like cells, such as presence of calponin^+^ CAF-like cells concomitant with absence of αSMA^+^ CAFs (patients #1,2) or predominance of αSMA^+^ CAFs in parallel with a negligible number of calponin^+^ CAF-like cells (patient #3) may suggest molecular/phenotypical modifications in these stromal cells as a factor of the activity of pembrolizumab, which subsequently could reflect different trends of activity. For example, it has been reported that the microenvironment of normal prostate comprises calponin^+^ smooth muscle cells that maintain differentiation of adjacent epithelial cells and inhibit their proliferation, while reciprocally, the epithelial cells maintain the smooth muscle phenotype of the stromal cells [23]. In contrast, the neoplastic TME of prostate cancer is predominated by αSMA^+^ CAFs with a negligible number of calponin^+^ smooth muscle cells. The interactions of αSMA^+^ CAFs and calponin^+^ CAF-like with the tumor cells in OSCC patients treated with pembrolizumab as well as the clinical effect of their different phenotypes should be further investigated.

In summary, although we are only at the beginning of the immunotherapy era for head and neck/OSCC, encouraging results have started to emerge from the few controlled clinical trials using checkpoint inhibition of the PD-1/PD-L1 pathway [12]. Stratification of patients eligible for this new treatment modality is nowadays based only on the clinical stage and the PD-L1 combined score of >1. Attempts to predict responsiveness to treatment comprising molecular/cytogenetic signatures based on tumor features prior to treatment, are underway. We have characterized specific populations of immune-related cells and CAFs after treatment with pembrolizumab, which highlighted several aspects of the tumor-TME interactions that have taken place as a result of drug administration. The potential associations between microscopical and molecular findings and clinical outcomes should be examined in larger samples of patients after accumulation of substantial clinical data and follow-up examinations.

## Data Availability Statement

The original contributions presented in the study are included in the article/supplementary material, further inquiries can be directed to the corresponding author/s.

## Ethics Statement

The studies involving human participants were reviewed and approved by IRB of Sheba Medical Center, Tel Hashomer. The patients/participants provided their written informed consent to participate in this study.

## Author Contributions

AD and MV: conceptualization, methodology, and writing—original draft preparation. AD, MV, IG, EA, IB, and RY: investigation and writing—review and editing. IG and IB: resources. MV and IG: supervision. All authors have read and agreed to the published version of the manuscript.

## Conflict of Interest

The authors declare that the research was conducted in the absence of any commercial or financial relationships that could be construed as a potential conflict of interest.
